# Construction of Prediction Model of Renal Damage in Children with Henoch-Schönlein Purpura Based on Machine Learning

**DOI:** 10.1155/2022/6991218

**Published:** 2022-05-23

**Authors:** Tingting Cao, Ying Zhu, Youyu Zhu

**Affiliations:** ^1^Department of Dermatology, Anhui Provincial Children's Hospital, Hefei 230051, China; ^2^Department of Nephrology, Anhui Provincial Children's Hospital, Hefei 230051, China; ^3^School of Basic Medical Sciences, Anhui Medical University, Hefei 230032, China

## Abstract

**Objective:**

The children with Henoch-Schönlein purpura (HSP) may suffer from renal insufficiency, which seriously affects the life and health of the children. This study aims to construct a prediction model of Henoch-Schönlein purpura nephritis (HSPN).

**Methods:**

A total of 240 children with HSP treated in dermatology and pediatrics in our hospital were selected. The general information, patients' clinical symptoms, and laboratory examination indicators were collected for feature selection, and the XGBoost algorithm prediction model was built.

**Results:**

According to the input feature indexes, the top ten crucial feature indicators output by the XGBoost model were urine N-acetyl-*β*-D-aminoglucosidase, urinary retinol-binding protein, IgA, age, recurrence of purpura, purpura area, abdominal pain, 24-h urinary protein quantification, percentage of neutrophils, and serum albumin. The areas under the curves of the training set (0.895, 95% CI: 0.827-0.963) and test set (0.870, 95% CI: 0.799-0.941) models were similar.

**Conclusion:**

The prediction model based on XGBoost is used to predict HSP renal damage based on clinical data of children, which can reduce the harm caused by invasive examination for patients.

## 1. Introduction

Henoch-Schönlein purpura (HSP) is one of the most common systemic vasculitides in childhood, a common vascular allergic disease. It mainly affects the skin, kidneys, intestines, joints, and other body parts [1]. In recent years, the number of children with HSP has increased significantly, and some studies show that the annual incidence of HSP is 160-191 cases per million children [2]. HSP points to the body receiving the stimulation of all kinds of sensitizing material, bringing about capillary brittleness and permeability enhancement inside the body, and causing inflammation or bleeding in the place such as skin, joints, and bowel [1, 3]. Clinical features of Henoch-Schönlein purpura nephritis (HSPN) were the fibrosis in patients with renal fibrosis [4]. HSPN is the most common secondary glomerular disease in children [5, 6].

Epidemiology suggests that HSP patients develop HSPN at a rate as high as 30% to 50% [7]. Although most HSPN patients have a good prognosis, 1%-3% of the children still suffer from renal insufficiency to end-stage renal failure, which seriously affects the life and health of the children [8]. Therefore, an early and accurate diagnosis of HSPN is crucial for prognosis and individualized treatment. Kidney biopsy is the gold standard for the diagnosis of HSPN. Still, this method is invasive and difficult for parents and children to accept, leading to some patients with severe kidney disease at the time of diagnosis [9].

Machine learning can use clinical data to build a prediction model and verify its predictive efficiency [10–12]. In recent years, the application in the medical field has been increasing gradually [13–16]. To our knowledge, there are few studies on machine learning to predict HSPN. Therefore, this paper mainly constructed a prediction model based on machine learning to predict the occurrence of renal damage in HSP through clinical data, providing a new method for the efficient diagnosis of HSPN in children diagnosed with HSP for the first time in dermatology.

## 2. Methods

### 2.1. General Information

A total of 240 children with HSP treated in dermatology and pediatrics in our hospital from October 2019 to December 2021 were selected, of which 153 were complicated with HSPN. According to the European Union Against Rheumatism [17], HSP is diagnosed as a palpable rash (essential) with at least one of four clinical symptoms: Abdominal pain, arthritis or arthralgia, renal involvement, and histopathological findings suggest IgA deposition. Renal impairment was predominantly clinical: abnormalities in hematuria, proteinuria, and renal function, such as increased serum creatinine (SCr) and decreased estimated glomerular filtration rate (eGFR), within 6 months of the course of HSP. The calculation formula of eGFR is as follows: ≤16 years old using Schwartz formula [18]; CKD-EPI formula was used when >16 years old [19]. When the eGFR <90 ml/(min·1.73 m^2^), it is considered as renal insufficiency.

### 2.2. Predicted Index

The indicators tested in this study mainly include general information, clinical symptoms, and laboratory indicators. General information includes sex, age, and season of onset. Clinical signs and symptoms include joint swelling, abdominal pain and gastrointestinal bleeding, purpura of the upper body skin, and recurrence of purpura. Laboratory indicators include blood routine tests, urine routine tests, and biochemical tests.

### 2.3. Machine Learning

The machine learning used in this study is the integrated machine learning XGBoost algorithm based on a classification and regression tree [20]. XGBoost algorithm has high scalability and high computing speed. Under the same environment and conditions, the XGBoost algorithm is more than 10 times faster than similar algorithms [21]. The specific detection process is shown in Figure 1.

XGBoost is an ensemble learning algorithm based on gradient boosting. Its principle is to achieve an accurate classification effect through the iterative calculation of a weak classifier [22]. It is an additive expression consisting of *K* base models:

(1) $$\begin{array}{c} \hat{y_{i}}=\overset{k}{\underset{t=1}{\sum }}f_{t}\left(x_{i}\right), \end{array}$$

where *f*_*t*_ is *k* basis models and $\hat{y_{i}}$ is the predicted value of the *i*th sample.

The model's deviation and variance jointly determine the model's prediction accuracy, and the variation of the model is embodied as the loss function. Therefore, the objective function is composed of the model's loss function and the regular term *Ω* that inhibits the complexity of the model. Thus, the objective function can be expressed as

(2) $$\begin{array}{c} \text{obj}=\overset{n}{\underset{i=1}{\sum }}l\left(y_{i},{\overset{\wedge }{y_{i}}}^{t}\right)+\overset{k}{\underset{t=1}{\sum }}\Omega \left(f_{t}\right). \end{array}$$

According to the calculation method of the Taylor formula, the above objective function can be written as

(3) $$\begin{array}{c} \text{ob}{\text{j}}^{\left(t\right)}=\overset{n}{\underset{i=1}{\sum }}l\left(y_{i},{\overset{\wedge }{y_{i}}}^{t}\right)+\overset{k}{\underset{t=1}{\sum }}\Omega \left(f_{t}\right)=\overset{n}{\underset{i=1}{\sum }}l\left(y_{i},{\hat{y}}_{i}^{t-1}+f_{t}\left(x_{i}\right)\right)+\overset{t}{\underset{i=1}{\sum }}\Omega \left(f_{i}\right). \end{array}$$

The CRT is defined as *f*_*t*_ = *w*_*q*_(*x*), *x* is a certain text, *q* (*x*) represents the leaf node where the sample is located, and *w*_*q*_ represents the value of the leaf node *w*. Therefore, *w*_*q*_(*x*) represents the value of *w* of each sample (i.e., the predicted value). The regular term of the objective function can be defined as

(4) $$\begin{array}{c} \Omega \left(f_{t}\right)=\lambda T+\frac{1}{2}\lambda \overset{T}{\underset{j=1}{\sum }}w_{j}^{2}. \end{array}$$

Gradient enhancement generates a series of CRTs in the training process. The corresponding value of the leaf node of the CRT is an actual score, and the cumulative score of each CRT is the final predicted value. We test the accuracy of the algorithm using the 5-fold crossover method. The data set was divided into five parts, 4 of which were taken as the training set and the other as the test set. The accuracy of each experiment was obtained, and the average accuracy of the 5 results was taken as the estimation of the algorithm's accuracy. The specific modeling process is shown in Figure 2.

### 2.4. Statistical Analysis

Counting data were counted by *χ*^2^ test. Measurement data were expressed by mean ± standard deviation and *t* test was adopted. *P* < 0.05 means the difference is statistically significant.

## 3. Results

### 3.1. General Information

Among the 240 children with HSP, there were 126 males and 114 females. The onset age was 2-16 years old, with an average age of 9.03 ± 2.68 years old. Among them, 62 cases (25.8%) occurred in winter, 102 cases (42.5%) had joint swelling and pain, 128 cases (53.3%) had abdominal pain and gastrointestinal bleeding, and 38 cases (15.8%) had upper body skin purpura. There were 153 cases of HSPN children and 87 cases without renal damage. There was no significant difference between the training group and the test group in gender, onset season, joint swelling and pain, abdominal pain, purpura of the upper body, and HSPN (Figure 3, *P* > 0.05).

### 3.2. Selection of Predictive Features

According to the statistical analysis results, gender is an insignificant factor in predicting the occurrence of HSPN in general information. The indicators of clinical symptoms are all statistically significant (*P* < 0.05) (Table 1).

The correlation of HSPN occurrence was predicted according to laboratory indexes such as biochemical tests, among which there was no significant difference in HSPN in platelet count, C-reactive protein, total cholesterol, IgM, and D-dimer (*P* > 0.05) (Table 2). However, the other indexes including white cell count, percentage of neutrophils, percentage of eosinophil, serum albumin, serum creatinine, IgG, IgA, IgE, hospitalization time, rinary retinol-binding protein (RBP), urine N-acetyl-*β*-D-aminoglucosidase (NAG), and 24-h urinary protein quantification were significantly correlated with HSPN (*P* < 0.05).

### 3.3. Prediction Results of XGBoost Algorithm Model

The XGBoost model automatically calculates features. According to the input feature indexes, the top ten important feature indicators output by the XGBoost model are as follows (Figure 4): NAG, RBP, IgA, age, recurrence of purpura, purpura area, abdominal pain, 24-h urinary protein quantification, percentage of neutrophils, and serum albumin.

### 3.4. Performance Evaluation of Model Prediction

In the training set, the area under the curve of the XGBoost model was 0.895 (95% CI: 0.827-0.963). In the test set, the area under the curve of the model was 0.870 (95% CI: 0.799-0.941). The XGBoost prediction model has good sensitivity and specificity. The receiver operation characteristic curves of XGBoost algorithm model is shown in Figure 5.

## 4. Discussion

HSP is a kind of systemic vasculitis, which mainly involves the skin, joints, gastrointestinal tract, capillaries, and small blood vessels of the kidney, accompanied by significant deposition of IgA [23]. Clinically, it is more common in children. It has been reported that more than 90% of HSPN occurs in children and adolescents, accounting for the first place in children with secondary nephropathy. Kidney biopsy is invasive and difficult for parents and children to accept [9]. Therefore, we predicted the incidence of HSPN from clinical data, clinical symptoms, and laboratory test indicators based on the XGBoost prediction model.

The XGBoost model can automatically obtain the importance score of each attribute, thus effectively filtering features. Our study screened children for general information, clinical symptoms, and laboratory test indicators. The top 3 indicators based on the XGBoost model are NAG, RBP, and IGA. Our results are consistent with Karadag et al. [24], who believe that vascular endothelial injury was an essential link in the pathogenesis of HSP. The possible reasons are as follows: (1) The permeability of the tube wall increased due to allergic reaction, and extravasation increased the concentration and slowed the blood flow. In a high viscosity state, immune complexes were more likely to deposit, further damaging the vascular endothelium and increasing the chances of platelet counting adhesion and self-aggregation. (2) Inflammatory reaction damages vascular endothelium. The damaged vascular endothelium enhances the coagulation promoting effect, stimulates the release of platelet count activating factor, and further promotes the activation and adhesion of platelet count.

Serum IgA is the main component of the body's mucosal defense system. It is widely distributed in milk, saliva, and mucosal secretions of the gastrointestinal tract, respiratory tract, and urogenital tract. Therefore, it plays a vital role in the first line of defense against infection, especially in the respiratory tract and intestinal tract. This is also an essential indicator in the prediction model of this paper. NAG is a lysosomal enzyme that occurs in the urinary system and is usually found in very low levels of urine. When the tubular cells are damaged, many NAG is released from the tubular epithelial cells into the urine, where NAG levels are elevated. RBP is the third important feature in the prediction model in our study. Liu et al. believed that the RBP has an important predictive value for delayed renal involvement in children with HSP [25].

In this study, the prediction model constructed based on the XGBoost algorithm can effectively reduce the overfitting problem and automatically specify the default branch direction for missing values, thus improving the algorithm's efficiency [26, 27]. Therefore, this provides more possibilities for the extensive application of the model. In addition, the areas under the curves of the training set (0.895, 95% CI: 0.827-0.963) and test set (0.870, 95% CI: 0.799-0.941) models are similar and have good sensitivity and specificity. Thus, the prediction model based on XGBoost can provide a new method for diagnosing HSPN in children diagnosed with HSP for the first time in dermatology.

There are several limitations to our study. It was a single-center retrospective study with a small sample size and no external validation. Secondly, due to the limitation of data sources, although this study included many predictive variables for screening, it was still not comprehensive. There may be potential predictive variables that were not included. In addition, this will further limit the advantage of the XGBoost algorithm. The next study will increase the sample size and expand the prediction index.

## 5. Conclusion

Based on the XGBoost prediction model, we can preliminarily predict HSP renal damage according to clinical test data in dermatological outpatient work. This can reduce the harm caused by invasive examination of children. It provides a new idea for the prognosis of children with Henoch-Schönlein purpura in the first diagnosis of dermatology. In future work, we will improve the shortcomings, starting from clinical needs, to better serve the clinical application.

## Figures and Tables

**Figure 1:** Flowchart of XGBoost detection.

**Figure 2:** Modeling flowchart of XGBoost algorithm.

**Figure 3:** Comparison of clinical data between the training set and test set. There were no significant differences between training set and test set in gender (a), painful swelling of joint (b), season of onset (c), abdominal pain (d), purpura of upper body (e), and HSPN (f).

**Figure 4:** Ranking of important features of XGBoost model output.

**Figure 5:** The receiver operation characteristic curves of XGBoost algorithm model. (a) Training set. (b) Test set.

**Table 1:** Test results of general information and clinical symptom indexes.

Indexes	*χ* ^2^	*P*
*General information*		
Gender	0.038	0.758
Age	385.874	<0.001
Season of onset	8.983	0.009
*Clinical symptom*		
Abdominal pain	4.213	0.023
Painful swelling of joint	7.896	0.014
Purpura area	238.705	<0.001
Recurrence of purpura	7.942	0.012

**Table 2:** Test results of biochemical laboratory indexes.

Indexes	*t*	*P*
White cell count	-4.763	0.019
Percentage of neutrophils	1.684	0.041
Percentage of eosinophil	3.980	0.027
Platelet count	-1.415	0.185
C-reactive protein	0.970	0.384
Serum albumin	-4.542	0.021
Serum creatinine	-3.425	0.032
Total cholesterol	-0.468	0.571
D-dimer	-1.538	0.214
IgG	-3.978	0.030
IgA	-2.342	0.034
IgM	0.795	0.436
IgE	3.012	0.028
Hospitalization time	2.031	0.037
Urinary retinol-binding protein	-5.784	0.014
Urine N-acetyl-*β*-D-aminoglucosidase	3.869	0.028
24 h urinary protein quantification	4.825	0.024

## Data Availability

The data used to support the findings of this study are available from the corresponding author upon request.
